# FEA Simulation of the Biomechanical Structure Overload in the University Campus Planting

**DOI:** 10.1155/2020/8845385

**Published:** 2020-11-23

**Authors:** Stanislau Dounar, Alexandre Iakimovitch, Katsiaryna Mishchanka, Andrzej Jakubowski, Leszek Chybowski

**Affiliations:** ^1^Belarusian National Technical University, Nezalezhnosti 65, 220027 Minsk, Belarus; ^2^Maritime University of Szczecin, Waly Chrobrego 1-2, 70-500 Szczecin, Poland

## Abstract

Research of breakage of the chestnut tree branch on the planting of university campus is provided. Collapse is caused by a severe accidental wind gust. Due to collapse in the student environment, the investigation has additional methodical value for the teaching of FEA simulation. The model includes roots, trunk, branch, and conditional crown, where the trunk-branch junction is steady enough. The load-bearing system of tree is taken as an example of an effective bionic design. The branch has grown with the implementation of the idea of “equal-strength console”—the change of sections along the branch provides constant stress level and near uniform dispensation of their without stress concentrators. Static simulation of the tree loading is provided both in the linear formulation and in the geometrically nonlinear one. It is proved that in the trunk-branch junction area the stresses are twice lower than the branch itself, and it is not the place for fracture. For the given wind pressure, the work stress in the branch has exceeded twice the allowable level under bending with some torsion. In such construction (of the tree), the breakage could happen even in the perfect branch condition due to her severe overloading.

## 1. Introduction

The work relates to the sphere of the simulation (CAE) by the finite element analysis (FEA) [1, 2]. An investigation is close to the biomechanics [3, 4] because the stress-strain state of the tree branch and trunk is discussed [5]. The work focuses both on engineering situation of tree load-bearing system [6] and on the methodical use of the results to teach students the possibilities of bionic design [7] and creative problem solving [8].

On the border of the university campus of BNTU, there is a group of trees (Figure 1). This is part of a two-row planting, namely, chestnuts (*Aesculus hippocastanum*). The object of modeling is tree 1, whose huge branch collapsed on a windy day, causing material damage [9]. Breakage took place in the healthy, quality wood grains (fibers) in the area of the trunk-branch junction. The tree remains standing and continues to grow (Figure 2).

The branch had a developed crown opposing the wind, but there was no storm in the summer city. According to the weather station (located 5 km from the campus), the wind speed was only 12 m/s. Weather is regarded stormy if the wind speed exceeds 15 m/s.

University authorities decided to investigate the incident from an engineering point of view. Two groups of specialists were formed: experts in the field of computational flow dynamics (CFD-group) and analysts of load-bearing systems (stress analysis group (SA-group)) [10, 11].

The CFD-group has provided computer simulation of airflows nearby the tree (0.3 km vicinity [12]) and revealed strong local wind amplification. It turned out that the tree is placed in the focus of the double-wedged air manifold. The slot between buildings is continued by the gap in the double-row planting just before the tree. In sum, north-east wind is speeding up above university stadium and creates in the manifold stormy flow with the velocity of 24–25 m/s. Post factum observations of such local wind flow point out of its steady character—wind gusts last about 5–7 s without significant oscillations. Therefore, trees are bent in the near static mode.

The SA-group has simulated the tree as a load-bearing system standing under wind pressure [13]. The pressure value was extracted from CFD-group work results—normal level is equal (*p*_norm_^wind^ = 380 Pa). A wind pressure of 600 Pa was taken into account too, as possible limit level for hurricane-like situation. With the aim to disclose stress-strain state of the tree and to reveal issues of the breakage, the FEA was accomplished by the SA-group.

Simulation has shown interesting result in two directions: the engineering of biomechanical load-bearing system and the methodical improvement of teaching students the FEA.

## 2. Geometry Model of the Tree Load-Bearing System

### 2.1. Geometry Representation

The tree with a broken branch was both laser scanned and sketched by gardeners just after the breakage. The SA-group members have provided 3D-modeling of this tree to bring variability of shapes and reduce subjectivity of simulation (Figure 3). The scope of simulation embraces tree's trunk 1, huge branch 2, and crown. Remained branches 3 and 4 are not included in the simulation scope. They are shown as conditionally trimmed. Branches 5 and 6 hold the crown.

According to the idea of tree crown variability [14], just two crowns were imaginarily matched to a given tree. A freely growing crown in the curled version is shown in Figure 3(a) (CurlCrown; blown surface—51 m^2^). The crown grown in the constrained conditions (neighboring trees) has been built in the rectangular version in Figure 3(c) (RectCrown; blown surface—30 m^2^). Both types of crowns reach a height of 14 m. The main technic of 3D-building was surface pulling on by sections. There were 5 sections for the trunk. Section dimension changes from Ø580 mm to Ø390 mm going from the ground to the trimming level.

The branch is pulled on by four basic diameters (marks 2–5 in Figure 4(a)) from Ø380 to Ø240 mm. The height difference between point 2 and point 5 is equal to 4 m. Branch bend in the 3–4 span has a radius of 2.4 m. The branch moves away from the trunk at the 60° angle (mark A60 in Figure 4(b)). Trunk-branch junction is smoothed by fillet with 70 mm radius.

Model DoubleTree (Figure 4(c)) with two main branches, two crowns, and common trunk with roots was built for additional proving of simulation results.

### 2.2. Wood Material Models

For results of stability proving, three material models were accepted for a parallel manner using during simulation. It should bring more confidence in results and limit model uncertainties of all issues. In the first model (ChestISO), wood is considered an isotropic, fully elastic material obeying Hooke's law. According to the construction codes and sources [15], for the chestnut wood, it was appointed: the elastic modulus (*E* = 8000 MPa), Poisson's ratio (*μ* = 0.42), density (*ρ* = 600 kg/m^3^), and allowable stress (*σ* = 16 MPa) (it is taken the same both for tension and compression). As it is not reliable initial data about mechanical characteristics of the crown, they are appointed a little arbitrary. Crown rigidity is considered very low, i.e., elastic modulus (*E* = 2 MPa). Crown density is the variable parameter to simulate different mass of leaves on the branches (see below).

Orthotropic representation of the chestnut wood is provided in the parallel manner with the isotropic one. Model ChestTKP is based on the local civil engineering code [16]. Elasticity modulus along grain is taken 8000 MPa, transversal to grain (400 MPa) (no difference between radial and tangential direction) and shear modulus (all three) (400 MPa), and Poisson's ratios should be taken as 0.5, 0.02, and 0.02 (XY, YZ, and XZ instances).

Other orthotropic model ChestWH is more detailed and scientific [16, 17]. Elasticity modulus along grain is equal 9400 MPa, transversal to grain (358 MPa and 678 MPa) (radial and tangential direction), shear modulus (all three) (544 MPa, 396 MPa, and 134 MPa). Poisson's ratios should be taken as 0.495, 0.052, and 0.035 (XY, YZ, and XZ instances). Thus, using of three different models proves natural scattering of wood properties while simulating.

### 2.3. FEA Mesh Variations

Several FEA mesh models of different structure were created for tree simulation. Looking ahead, note all of them have shown good correspondence in results and minimal level of computing artefacts.

Objects named solids and parts are used in the meshing procedure. Solid brings monolithic mesh. The part consists of several solids touching each other. Mesher joins their local meshes by common nodes. So part mesh is one-piece too. Other variants to simulate interaction between solids or parts contact pair creation (special surface elements on the interface). For that work, contact pairs are always in the bonded state. They work as perfect thin rigid glue layers.

One of the finite element meshes is shown in Figure 5 (name it R-mesh (rare element density)). Finite elements have mostly tetrahedral shape. It relates to trunk 1 (Figure 5(c)) and to junction 3 between trunk 1 and branch 2. The branch itself is meshed by hexahedral elements. It brings better accuracy in the critical part of the model. At the same time, higher smoothness of the stress fields is achieved. The trunk and branch create single solid. Accordingly, the trunk's mesh 1 (Figure 5(c)) permanently transforms into the branch's mesh 2. For all wood, massive finite elements are joined together by common nodes. The tree's crown was represented by a separated mesh of volume finite elements. Crown and tree meshes were conjugated by contact pair.

Figure 6 depicts alternative mesh (D-mesh (finite element packed with higher density)). The trunk and main branch were split to the sets of small solids. It was done by planes normal to trunk/branch axes of growing. Solids 1 and 3 belong to the part “Branch.” Such solids are joined together by common nodes at the faces like 2 and 3.

Solid 4 and underlying ones create monolithic part “Trunk.” Parts “Trunk” and “Branch” are glued (BC) by bonded contact pair. Stress state for this model is shown in Figure 6(b). Stress field near marker BC is smooth and continuous. Also, interfaces between solids are not visible anywhere. It means precision and fidelity of the D-mesh model.

Mesh in Figure 6 is denser compared with one in Figure 5. Outer surfaces of the trunk and branch are covered in Figure 6 by set of thin finite element layers (3). It brings accuracy for representation of surface stress effects. Branch core is modelled relatively coarse finite elements (2). That is a standard FEA approach, especially that bending domination is expected. Line 2–2 (Figure 6(b)) goes between tension and compression zones. Equivalent stress maximum (34.529 MPa) here (D-mesh) relates well to analog simulation by R-mesh. Thus, both mesh models are appropriate enough.

### 2.4. Boundary Conditions

The simulation was provided in the static form. That assumption is based on the CFD-group conclusion as about smooth, long-time patterns of wind gusts in the local natural manifold acting on the simulated tree. Oscillations and resonant effects are out of modeling scope.

Crown is a conditional object of the plate's shape. Simulation has focused on the lower branch (1st order branch—cite of breakage). Branches of the 2nd order are placed above and are built approximately. Branches of the 3rd order are not regarded.

Interaction between crowns is not simulated. Leaves are considered inner components of the crown. The mass of all leaves on the main branch (crown mass) is a really uncertain parameter. It was taken at three levels—750, 1225, and 1550 kg—marked below as L-leaves, M-leaves, and H-leaves. Crown mass governs the gravity force. Simulation pointed out that gravity force starts to play a role only at hurricane-like wind pressure (600 Pa), where strong sloping of the crown occurs (Figure 7(c)).

The ground is simulated as a rigid base (mark A in Figure 7(a)). Wind pressure (mark B) is uniformly distributed upon the windward side of the crown. Gravity force (mark C) is dispensed through all materials according to their densities.

Parallel modelling by different models and various conditions is the feature of that work. Intentional variation of model factors was provided by different authors to control uncertainties. The aim of parallel simulations was to ensure result stability and to estimate the sensibility of tree stress-strain state to the chatter of the entering factors.

Table 1 depicts the scope of varied factors. Near full crossing of all steps was achieved. Geometrical linearity/nonlinearity of the tree model was investigated. That is a single kind of nonlinearity into the FEA model. Friction is not included, and wood is taken as fully elastic.

If the model was simulated as linear (Lin), only one step of loading is provided. The model undergoes stepped loading (30 steps) when large deformations are counted in the stiffness matrix of the tree, so geometrical nonlinearity (NonLin) became observable.

Variations during tree simulation pointed out two representative sets of boundary conditions. They are called “Light” (LiBC) and “Heavy” (HeBC) and are marked by color in Table 1. “Fork” space creates between them for other variants of the model parameters. LiBC set refers to the simple, isotropic, linear model of the tree under storm-like wind pressure. HeBC set gives possibility to estimate ultimate deflection of the heavy orthotropic tree in the near hurricane situation.

### 2.5. Nonlinearity and Orthotropy Checks

Meshes R-mesh and D-mesh were used for simulation as three wood material models. Loading was provided up to 600 Pa wind pressure. It was revealed (Figure 8(a)) that large deformation simulation (NonL) brings higher levels of stresses and displacements in the tree compared to geometrically linear model (Lin). Nonlinear solution points out rise of branch top displacement on 33%. Maximal equivalent stress rises on 35%. It relates to the tree with the heavy crown (H-leaves). In the case of light crown (L-leaves), the nonlinear curve passes lower. Here, the difference between nonlinear and linear results does not exceed 18%. It is obvious that deflection of heavy crone by wind stimulates growing of the gravity force moment. So, crown hanging-off additionally grows. Nonlinear simulation is the way to disclose that interaction.

The comparison of curves for the isotropic wood model (“ISO”) and orthotropic models (“TKP” and “WH”) is given in Figure 8(b). Orthotropic lines are placed near each other with the difference below 7%, whereas the isotropic model turns up much more rigid. Displacements for TKP-tree are 58% stronger than those for the ISO-tree (both models possess the same elasticity modulus at 8000 MPa).

However, stress levels for all three materials are placed in vicinity to each other (with the range of only 13%—despite of displacements). It relates to the nonlinear simulation of heavy crown trees.

In the “light-crown” case, wood material variation causes a difference of 15% for displacements and 6% for stresses (linear solutions).

As a result, there are no principal differences between linear and nonlinear solutions concerning the shape of deflection and stress state features.

## 3. Results and Discussion

### 3.1. Depiction of the Tree Stress-Strain State for Isotropic Model

Figure 9(a) shows natural scale deformational displacements of the tree. The crown significantly deflects on its top (above 2 m). The branch is much more rigid, and the displacement (below the crown) is less than 100 mm.

The distribution of the equivalent stress (*σ*_*e*_) for the DoubleTree model is smooth enough (Figure 9(b)). There is not just local, sharp stress concentration. The trunk is stressed moderately (14.5 MPa). Some stress increasing is visible at the trunk-root junction (29.6 MPa). The main attention should be paid to the strips “34.448 MPa” and “34.077 MPa.” The first marker precisely relates to the place of the branch breakage.

Figure 10 depicts the concentration of equivalent stress (*σ*_*e*_) (von Mises stress) in the basic tree model, which discloses both one-axis tension regions (indicates principal maximal stress (*σ*_1_)) and one-axis compression regions (principal minimal stress (*σ*_3_)). The tree surface has no local stress concentrators, discontinuities, and high-gradient regions. The bottom part of the branch is the only placed with relatively high stresses. Here, Strip of Strong Tension (SSTe) is shown (between marks 1–2 in Figure 10(a)), where equivalent stress reaches level *σ*_*e*_ = 34.181 MPa. This is the most tensioned part of the tree on the windward side far away from the trunk-branch junction—“tensioned fiber”—by a classic theory of bending. Equivalent stress (*σ*_*e*_) near the trunk-branch junction is equal only to 13.614 MPa. The trunk is a slightly stressed object with *σ*_*e*_ = 6.509 MPa.

Strip of Strong Compression (SSCo) lays between 3 and 4 in Figure 10(b). Equivalent stress (*σ*_*e*_) here reaches 34.08 MPa level. That is so-called “compressed fiber” by classic theory of bending.

Figure 11 demonstrates the direction of the principal stress vectors. On the leeward side, one could see dominance of the principal minimum stress (*σ*_3_) (blue arrows in Figure 11(a)) as manifestation of SSCo feature. On the windward side, we can see the principal maximum stress (*σ*_1_) (red arrows in Figure 11(b)) as SSTe feature. There are not visible green arrows, which means that the principal middle stress (*σ*_2_) is near zero in the whole tree. Therefore, exactly, SSTe is the place of one-axis tension, and at the same time, SSCo is the place of one-axis compression. Both *σ*_1_ and *σ*_3_ vectors are oriented along the branch. This is a clear picture of bending. Some vector's winding around the branch axis points out the presence of the small torsion moment (in a moderate proportion to the bending one).

The conclusion about bending dominance in the stress-strain state of the branch is proved by distributions of the principal stresses (Figure 12). The fields of tension on windward side are shown in Figure 12(a) (almost completely coincident with Figure 10(a)), where principal maximum stress (*σ*_1_) creates SSTe (marks “30.729”–“34.069”–“30.177”). It is the single place of high tension, but longitudinal gradients are very low here, because tension stress is near the same in it. Therefore, SSTe should be taken into account as ridge-like increase, not just a point of stress concentration, and wood breakage could start spontaneously in any place of SSTe.

The picture of the principal minimum stress (*σ*_3_) shows smooth focusing of compression with small gradients along the branch from leeward (marks “-31.058”–“-34.103”–“30.5” in Figure 12(b)) and points out the SSCo.

The SSTe and SSCo features received elongated shape. Large length is causes by branch section changing. The branch as the kind of beam very close to the ideal “equal-strength console” is rising in diameter from leaves to the trunk. The bending moment is enhancing in this direction at the same time. Branch thickening (inertia moment enhancing) effectively counteracts to growing bending moment. The quick increase of branch diameter in the trunk vicinity is relating the reinforcement of the trunk-branch junction. It results in stresses stabilizing and is an example of self-organized wood growth to limit and level the stresses. This is the bionic stresses stabilization (BiSS) or “ironing” of stress concentrators.

### 3.2. Stress Distribution for Orthotropic Wood Model

Wood grain (fiber) orientation is always known for a living tree only approximately. Thus, three simple, different variants of orientation were simulated (Figure 13) on the D-mesh base. It is a geometrical model assembled from split solids. Wood grain vector (WGV) was oriented inside every solid normally to its bottom face. It caused (Figure 13(a)) an uneven shape of stress isolines. Transitions between solids are clearly visible.

Nevertheless, stress picture, described above for the isotropic model (Figure 10(b)), is preserved. One can see stress concentrator (SSCo), marked as A (38.24 MPa). Additionally, two local extremums (B: 25.27 MPa) and (C: 24.58 MPa) are founded at ends of branch-trunk junction.

The system consisting of stress spots A, B, and C is revealed again in Figure 13(b) (vertical-dominant orientation of WGV) and in Figure 13(c) (WGV orients along the branch and smoothly extends that orientation into the trunk).

It may be stated that the orthotropic model of the tree is more tangible to local geometry unevenness than isotropic one. Spots B and C probably are tied with some kind of that effect. Orientation vector variations are not crucial for the stress state of a tree branch. Main stress spots and stress levels remain the same for both isotropic and orthotropic wood material representations.

### 3.3. Nonlinear Estimation of the Branch Overloading

The stress-strain state pictures, shown above, point out that branch breakage under wind pressure (*p*_norm_^wind^ = 380 Pa) is highly likely possible. Nonlinear geometry effects amplify deformation and overloading of the branch through displacing of the crown's mass center to leeward. In its turn, the gravity force starts to create a bending moment relative to the trunk's rest (eccentrically compression) and increase even more deviation of the branch from the vertical axis.

The comparison of the linear and nonlinear solutions is given in Figure 14.  Figure 14(a) shows the picture of equivalent stress (*σ*_*e*_), calculated for fully linear assumptions and one-step loading.  Figure 14(b) gives the distribution of equivalent stress, when the large deformation effects are accounted and the stepped loading solution is achieved. In the second case, the crown's top displacement has risen about twice. The stresses along SSTe and SSCo have grown approximately in a quarter. Equivalent stress on the windward side of the branch (SSTe) is increasing from 54.2 MPa (Figure 14(a)) to 67.1 MPa (Figure 14(b)). For the trunk part of the tree, the nonlinear effects are not so strong.

Thus, the pressure of a stormy wind overloads the tree branch up to fracture. It happens above the allowable stress level for wood. Therefore, there is no need to look for a concentrator or damaged place along the branch to explain the event of destruction [18]—the branch should fall under the influence of strong bending and torsion moments. Our task was to point out the fact of severe overloading in healthy wood material possibility, but details of the cracking model may be the topic for the further investigation [19–21]. In the future research, the uncertainty analysis is planned to be done [22, 23].

### 3.4. Variations for Sensitivity Checks: Stability of “Ironed” Stress Concentrators during Wind Rotation

The DoubleTree model (Figure 15) approves earlier conclusions. Both branches have ribbon-like tensed and compressed fields. Stress peaks are placed far enough from the trunk. The trunk itself is stressed stronger (*σ*_*e*_ = 14.57 MPa in Figure 15(d)) due to bigger blown surface of both crowns. It should pay attention to the underground stress concentrator (*σ*_*e*_ = 29.68 MPa) in Figure 15(c).

Wind direction influence on the branch stress-strain state is estimated in Figure 16. The tree crone is built as a kind of sail in that work. Four trees with identic, parallel crones were included in the model. Wind assumes acting normally to the flat crones.

Every trunk-branch system was rotated at its own angle around the vertical axis relative to the crone. The angle changes at 30° from tree to tree. So, left tree orientation (Figure 16) is similar to the one from Figure 10. Right tree (Figure 16) has accumulated an angle of rotation equal to 90°. Its loading represents blowing off from the perpendicular direction.

Four markers (34.13–34.48 MPa) show high independence of tension stress strips (SSTe) from the wind direction. Compression stresses (SSCo) from the other side of the branch are at the constant level too. Bending (paired tension – compression system) is the dominating feature of the branch stress-strain state. Some moderate torsion is present for every branch in Figure 16. Thus, even large changes in the wind direction remain, and the branch stress state is the same. The pair of ironed stress concentrators on the healthy branch should be taken as steady BiSS effect.

Let us pay attention to a whole lot of similar trees, planted in university campuses. Some of them need serious assessment and possibly help (Figure 17).

Each problematical tree is the object for FEA analysis. The simulation could predict eventual collapse. In addition, simultaneously, a lively and directly learning process the mechanical students may be provided. The spheres of 3D-scanning, recovery of geometry, dynamics of fluid, and 3D-printing may be involved.

## 4. Conclusions

The investigated branch during a storm undergoes mainly the bending and some torsion. Gravity compression does not take a significant part in the stress state.

The SSTe is formed on the windward side in the bottom third of the branch. On this level, on the leeward side, the SSCo is revealed. Both of the strips form a picture of bending of the console beam.

The branch is a beam similar to the ideal “equal-strength console.” The main stresses (*σ*_1_ and *σ*_3_) (values near the constant) appeared on the SSTe and SSCo along the branch. On those areas, it is not any stress concentrator, but the uniform stress state only. It is provided by spontaneous BiSS and effective self-reinforcement through the self-organized wood growth.

The trunk-branch junction is steady and developed. In the junction area, the stresses are twice lower than the branch itself. Thus, trunk-branch junction is formed as a region of the significant reinforcement, and it is not the place for fracture.

High stresses rising in a smooth and uniform manner only along SSTe and SSCo are reached at 30-34 MPa at the moderate crown (RectCrown model). But it significantly exceeds the allowable stress for chestnut wood (16 MPa). When the crown was developed (CurlCrown model), a tree deformation becomes nonlinear, and the stress at all rises up to 67 MPa due to partially eccentric action of the gravity force.

In such tree construction for the given wind pressure, the breakage of branch could happen even in the perfect branch condition and without the stress concentrator due to severe overloading, because the predicted stress exceeds twice allowable stress for the chestnut tree.

Inside almost every university campus, we can find appropriate plants and trees as the investigation object. Because the campus is a part of the student's environment, then modeling of the tree attracts interest of students. The load-bearing system of the tree serves as a complex and at the same time understandable example to study both FEA simulation and bionic principles of the design.

The tree branch became a good illustration of the “equal strength console” idea. We can see the rational changing of branch sections—stresses are leveled along the main part of the branch. It makes students see the bionic design sense.

Tree simulation teaches students to create models of load-bearing systems without stress concentrators. Mechanical students generally know that different junctions are usually the most stressed places into machines. The trunk-branch junction is the counterexample. It shows the potential of bionic-style reinforcements.

The task on tree theme teaches the students a lot of modeling technics. There are flexible system simulation, geometrical nonlinearity, and branch-crown contact interaction. Thus, student gets acquainted with the complex stress state of the branch, including bending, torsion, and eccentrical compression.

## Figures and Tables

**Figure 1:** The simulated tree (1) long before breakage of branch (2014).

**Figure 2:** The trunk-branch junction just after branch sawing (2018).

**Figure 3:** Tree geometry: (a) model with curled crown (CurlCrown) on the downwind side; (b) the internal dimensions of the branch; (c) elongated crown (RectCrown) from upwind.

**Figure 4:** Models of the branch: (a) the trunk-branch junction; (b) the tree with two branches; (c) two crowns and stylized roots (DoubleTree).

**Figure 5:** Meshes for: (a) leeward side of crown; (b) windward side of crown; (c) trunk 1 with junction 3 to branch 2.

**Figure 6:** Dense mesh for split solids (D-mesh): (a) partial view at solids; (b) picture of equivalent stress (*σ*_*e*_) (MPa) for LiBC condition set (stated below).

**Figure 7:** Tree fastened to ground A and loaded by B (wind pressure) and C (gravity force): (a) leeward windward; (b, c) windward. Deformation shapes and reaction force vectors are for LiBC and HeBC condition sets at (b, c), respectively: ×1.

**Figure 8:** Curves of “along-wind” crown top displacement (mm) (mark “C” in the curve name), branch top displacement (mark “B”), and maximal equivalent stress on the branch surface (10^−1^ MPa, mark “S”): (a) linear (“Lin”) and nonlinear (“NonL”) loading for the heavy (“H”) crown (means H-leaves) and for the light (“L”) one (means L-leaves) in the case of ChestWH material; (b) nonlinear tree loading for materials ChestISO, ChestTKP, and ChestWH (marks “ISO,” “TKP,” and “WH”, respectively); H-leaves: HeBC.

**Figure 9:** Total displacement (mm) of the tree with the crown of RectCrown type under wind pressure (*p*_norm_^wind^ = 380 Pa) (a) and the picture of equivalent stress (*σ*_*e*_) (MPa) for the DoubleTree model (b).

**Figure 10:** Distribution of the equivalent stress (*σ*_*e*_) (MPa) through the surfaces of the branch and trunk on the windward (a) and leeward (b) sides. Pressure (*p*_norm_^wind^) = 380 Pa; RectCrown, ×1.

**Figure 11:** Vectors of principal stresses on the leeward (a) and windward (b) sides. Pressure (*p*_norm_^wind^) = 380; RectCrown, ×1.

**Figure 12:** Distributions of the principal maximum stress (*σ*_1_) (a) from windward and minimum stress (*σ*_3_) (b) from leeward. Pressure (*p*_norm_^wind^) = 380 Pa; RectCrown, ×1.

**Figure 13:** Distributions of the equivalent stress (*σ*_*e*_) for different wood orthotropy models: “normal-to-split” wood grain (a), vertical-dominant wood grain (b), and “along main branch” wood grain (c). Pressure (*p*_norm_^wind^) = 380 Pa, leeward; (a, b) ChestWH and (c) ChestTKP; Lin; ×1.

**Figure 14:** Equivalent stress distribution (*σ*_*e*_) (MPa) for the linear solution (*a*) and for the geometrically nonlinear one (*b*; stepped loading). Peak wind pressure (*p*_peak_^wind^) = 600 Pa; ×1.

**Figure 15:** Simulation of the tree with two big branches (DoubleTree model and LiBC) loading by wind pressure (*p*_norm_^wind^) = 380 Pa: (a) double fastening root; (b) vectors of principal stresses; (c) principal maximum stress (*σ*_1_) (MPa); (d) equivalent stress distribution (*σ*_*e*_) (MPa); ×1.

**Figure 16:** Stability of peak stress (*σ*_1_) (MPa) on the branch regardless of the wind direction (from left to right, trunk rotates at angles 0°, 30°, 60°, and 90° relatively to crown). LiBC, ×1.

**Figure 17:** Obliquely growing campus tree in the need for assessment and FEA simulation.

**Table 1:** Steps of model factors to vary.

Model variation factors	Leading sets of boundary conditions (BC)		
	LiBC	HeBC	
Trunk-branch material	ChestISO (isometric)	ChestTKP (orthotr.)	ChestWH (orthotr.)
Mesh	R-mesh	D-mesh	
Crown shape	CurlCrown	RectCrown	DoubleCrown
Leaves mass	L-leaves (750 kg)	M-leaves (1225 kg)	H-leaves (1550 kg)
Wind pressure	380 Pa	600 Pa	
Geometrical nonlinearity	Lin (1 step)	NonLin (30 steps)	

## Data Availability

All results are provided in the paper.
